# Impact of magnetic immobilization on the cell physiology of green unicellular algae *Chlorella vulgaris*

**DOI:** 10.1080/21655979.2020.1718477

**Published:** 2020-01-29

**Authors:** Seyedeh-Masoumeh Taghizadeh, Aydin Berenjian, Kit Wayne Chew, Pau Loke Show, Hayyiratul Fatimah Mohd Zaid, Hamidreza Ramezani, Younes Ghasemi, Mohammad Javad Raee, Alireza Ebrahiminezhad

**Affiliations:** a Department of Pharmaceutical Biotechnology, School of Pharmacy and Pharmaceutical Sciences Research Center, Shiraz University of Medical Sciences, Shiraz, Iran; b School of Engineering, Faculty of Science and Engineering, University of Waikato, Hamilton, New Zealand; c School of Mathematical Sciences, Faculty of Science and Engineering, University of Nottingham Malaysia, Semenyih, Malaysia; d Department of Chemical and Environmental Engineering, Faculty of Science and Engineering, University of Nottingham Malaysia, Semenyih, Malaysia; e Fundamental and Applied Sciences Department, Centre of Innovative Nanostructures & Nanodevices (COINN), Institute of Autonomous System, Universiti Teknologi PETRONAS, Bandar Seri Iskandar, Malaysia; f Department of Medical Nanotechnology, School of Advanced Medical Sciences and Technologies, Shiraz University of Medical Sciences, Shiraz, Iran

**Keywords:** Aquatic ecosystems, ecotoxicity, magnetite, magnetic harvesting, mtt assay, nanosafety

## Abstract

Cell immobilization on the magnetic nanoparticles (MNPs) and magnetic harvesting is a novel approach for microalgal cells separation. To date, the effect of these nanoparticles on microalgal cells was only studied over a short period of time. More studies are hence needed for a better understanding of the magnetic harvesting proposes or environmental concerns relating to long-term exposure to nanoparticles. In this study, the impact of various concentrations of MNPs on the microalgal cells growth and their metabolic status was investigated over 12 days. More than 60% reduction in mitochondrial activity and pigments (chlorophyll a, chlorophyll b, and carotenoids) content occurred during the first 6 days of exposure to ≥50 µg/mL nanoparticles. However, more than 50% growth inhibitory effect was seen at concentrations higher than 400 µg/mL. Exposure to MNPs gradually induced cellular adaptation and after about 6 days of exposure to stress generating concentrations (˂400 µg/mL) of IONs, microalgae could overcome the imposed damages. This work provides a better understanding regarding the environmental impact of MNPs and appropriate concentrations of these particles for future algal cells magnetic immobilization and harvesting.

## 1. Introduction

Magnetic nanoparticles are among the nanomaterials that are commonly used in many different fields of modern technology such as targeted drug delivery, hyperthermia, magnetic resonance imaging (MRI), RNA and DNA purification, enzyme and protein immobilization, pathogen and nonpathogenic bacteria isolation and separation, environmental remediation, food industry, medical diagnostics, and cells harvesting [1–3]. Magnetic harvesting has opened a new avenue to functionalize, manipulation, and sedimentation of cells [4–7]. In a very recent short period of time, this novel approach was examined and employed to harvest a variety of cells, specially microalga as one of the most economical valuable cells [5,8–13].

For centuries, microalga was employed as a source of nutritional supplements, and in recent years, these cells were employed in technological process and production of bioactive materials such as pigments, amino acids, proteins, carbohydrates, sunscreen molecules, omega-3 fatty acids, antioxidants, and vitamins [14,15]. They are also employed as biofuel feedstock and refinement of polluted water by acting as a biologic filter for nitrogen, phosphorus, heavy metals, and toxic compounds [16–18]. While microalgae technology is growing by an astonishing rate, the cell harvesting is still the major challenge and a bottleneck in this industry. Microalga cells can be harvested by various techniques such as dewatering, flocculation, sedimentation, filtration, centrifugation, and magnetic harvesting [8,10]. Among these procedures, magnetic harvesting draws an increasing attention due to its simple operation, fast separation, low running cost, energy saving and nondestructive nature of employed magnetic fields [4,7].

This technique is based on the high affinity of the cell walls for adhesion to the inorganic compounds and surfaces. In fact, the cells are equipped with adhesion factors that help them to attach and colonize on the surfaces. During exposure to nanoparticles, adhesion factors make these particles attach and fill the cell surface with nanoparticles. Nanoparticles can also attach to the cells surface via nonspecific interactions such as hydrogen bonds, electrostatic, Van der Waals, hydrophobic, and hydrophilic forces [2,3,19,20]. The surface charge of living cells is negative and hence most experiments were performed by employing engineered magnetic nanoparticles with positive functionalities to provide more electrostatic attraction [9,12,13]. If magnetic nanoparticles attach on a particular cell in this order, the cell becomes magnetically responsive and can be easily manipulated using a magnet [9]. Due to the simplicity of operation facilities and required equipment and also the availability of giant powerful electrical magnets this technique can be scaled up easily.

In addition to facilitated harvesting, magnetic immobilization provides other advantages in biotechnological processes. It has been shown that magnetic nanoparticles may disrupt the cell membrane integrity and increase selective permeability of the membrane. Increase in membrane permeability results in facile mass transfer of nutrition and products and hence increases the cells performance [2,9]. This effect was also reported for magnetic modified microalga cells with high (over 95%) efficiency in cell recovery [11,13].

However, magnetic harvesting of microalgae has yet to be optimized and several key factors such as the effects of magnetic nanoparticles on growth, metabolism, and function of microalga cells need to be clarified. In several studies, different toxicity mechanisms were explained for magnetic nanoparticles. Due to the surface oxidation, these particles release iron ions that can catalyze the production of reactive oxygen species (ROS) in the Fenton’s reaction (equations 1 and 2) [21]. But, the toxicity of magnetic nanoparticles cannot be explained by purely chemical effects of the dissolved iron ions. There are particle-specific cytotoxic mechanisms which are due to stress or stimuli caused by the surface, size, and shape of the nanoparticles [22]. Furthermore, in the case of microalga, magnetic nanoparticles can reduce the light availability for the photosynthetic process [23].

(1) $$Fe^{2+}+\;H_{2}O_{2}\to \;Fe^{3+}+\;OH^{\cdot }+\;OH^{-}$$

(2) $$Fe^{3+}+\;H_{2}O_{2}\to \;Fe^{2+}+\;OOH^{\cdot }+\;H^{+}$$

*Chlorella vulgaris* is one of the most studied and known types of microalgae. This alga is used as the first choice in general experiments where we need a microalga model. Previous investigations revealed that magnetic nanoparticles have some toxic effects on *C. vulgaris* with deteriorative impacts on photosynthesis and proliferation. Also, oxidative stress was induced by these nanoparticles and the stress was in direct relation with the rate of metal ions release [24]. Nanoparticles coating has a significant role to control or even block the oxidative stress that is induced by magnetic nanoparticles. But, coating can magnify other deteriorative effect of nanoparticles such as indirect light shading effect due to nanoparticles colloid and direct shading effects due to cell agglomeration [25]. Previous experiments were performed for a time period of about 72-h of exposure to magnetic nanoparticles [24,25]. Meanwhile, in the magnetic immobilization setting, cells were exposed to magnetic nanoparticles for a long time period. On the other hand, there are no comprehensive data available about the impacts of magnetic nanoparticles on all biological and biotechnological aspects of *C. vulgaris* cells. To fill these data gaps, we evaluate the growth, metabolism (respiration and photosynthesis), and membrane integrity in magnetic immobilized *C. vulgaris* in contrast to free cells for a time period of 12 days. Also, these data are applicable for discussions about environmental contaminations with magnetic nanoparticles where these particles are released in soil and fresh water ecosystems.

## 2. Materials and methods

### 2.1. Preparation and characterization of MNPs

Magnetic nanoparticles (Fe_3_O_4_) with L-lysine coating were synthesized via copercipitation reaction of Fe^+2^ and Fe^+3^ in aqueous medium in the presence of L-lysine. In brief, 1.17 g of ferric chloride hexahydrate (FeCl_3_ · 6H_2_O) and 0.6 g of ferrous sulfate tetrahydrate (FeSO_4_ · 4H_2_O) (molar ratio 1.75:1, respectively) were dissolved in 50 mL deionized water and the mixture was stirred vigorously under N_2_ atmosphere at 70°C. After 30 min, 1.6 g of L-lysine were dissolved in 6 mL distilled water and rapidly added to the mixture and the reaction was stirred for another 30 min. Then, 5-mL NH_4_OH (32%) was added while the stirring was continued for 1.5 h. The sample particles were separated magnetically, washed with distilled water three times, and dried in an oven at 50°C overnight.

Sample particles were characterized by a Fourier Transformed Infrared spectroscopy (Bruker, Vertex 70, FT-IR Spectrometer), x-ray diffractometer (Siemens D5000), Vibrating Sample Magnetometery (VSM) (Meghnatis Daghigh Kavir Co., Iran), Differential Scanning Calorimetry (DSC) (BAHR Thermoanalyser DSC 302), and Transmission Electron Microscopy (TEM) (Philips, CM 10, HT 100 Kv).

### 2.2. Exposure of C. vulgaris to magnetic nanoparticles

A strain of *C. vulgaris* (MCCS 012) was employed in this experiment. The strain was identified by morphological characterizations and 18S rRNA gene sequencing. The DNA sequence is available in the NCBI under the accession number EU374170 [26]. The microalgal culture in BG-11 medium (5 × 10^6^ cells/mL) were exposed to 0, 12.5, 25, 50, 100, 200, 400, 600 and 800 µg/mL of magnetic nanoparticles (MNPs). Samples were incubated in a culture room under constant illumination (4150 lux) with a white fluorescent lamp at 25°C. The general morphology of *C. vulgaris* cells over 12 days of exposure to nanoparticles was evaluated by optical microscopy.

Interaction of magnetic nanoparticles with *C. vulgaris* cells was subjected to precise visualization by using electron microscopy. But there was a possibility for some nanoparticles to be unattached to the cells and float as free particles. To separate possible free particles from *C. vulgaris* cells, the samples were first subjected to mild centrifugation (2000 rpm for 2 min). But no significant nanoparticles were indicated in the supernatant and sudden sedimentation has occurred and resulted supernatant was completely clear. While presence of magnetic nanoparticles in colloidal form makes the suspension brown and turbid.

To prepare the samples for scanning electron microscopy (SEM) analysis, a thin smear of the cells was spread on the glass slide and dried at room temperature. The specimens were fixed by going through the fire of a Bunsen burner and set in 2.5% glutaraldehyde for 45 min. The slides were washed for 15 min in normal saline three times and dehydrated for 10 min at serial ethanol concentrations (30%, 50%, 70%, 80%, and 90%). Final dehydration stage was carried out for 20 min in absolute ethanol.

### 2.3. Direct cell counting

The growth characteristics of *C. vulgaris* in various MNPs concentrations were measured by direct counting method. Microalgal cells were enumerated using a Neubauer hemocytometer followed by staining with Lugols iodine solution (2%, v/v). Cell growth was determined at 3 days intervals over 12 days. Specific growth rate over 12 days was calculated according to equation (3).

(3) $$\mu =Ln\;\left(N_{2}-N_{1}\right)/\left(t_{2}-t_{1}\right)$$

where µ is the specific growth rate, N_1_ and N_2_ are the total cells/mL at day 1 (t_1_) and day 12 (t_2_) [1].

Percentage of growth inhibition (I%) was calculated according to equation (4).

(4) $$I\%\;=\;100*\left(\mu c-\mu \right)/\mu c$$

where µc is the specific growth rate of the control sample with no nanoparticles.

### 2.4. Mitochondrial activity

Mitochondrial activity of algal cells was evaluated via MTT (3-(4,5-dimethylthiazol-2-yl)-2,5-diphenyltetrazolium bromide) colorimetric assay at 3 days intervals. Reduction of the MTT to formazan was detected by color development at 550 nm. *C. vulgaris* cells were incubated in the presence of 4 mg/mL MTT at 37°C. After 3h, equal volume of DMSO was added and the samples were agitated vigorously and incubated at 37°C for 15 min to dissolve the formazan crystals. Samples were agitated again and absorbance was measured at 550 nm using an eppendorf BioPhotometer plus. The mitochondrial activity (M %) was calculated using the following formula.

$$M\%=\frac{At-Ab}{Ac-Ab}\times 100$$

where *A_t_, A_b_* and *A_c_* are the absorbance values of test, blank with no algal cell and control samples with no nanoparticle, respectively.

### 2.5. Chloroplasts activity

The effect of MNPs on the *C. vulgaris* chloroplasts was evaluated by chlorophyll and carotenoids assay. The content of chlorophyll and carotenoids were determined at 3 days intervals. Chlorophyll and carotenoids were extracted in methanol via the ultrasound-assisted extraction method [27].

### 2.6. Lipid content

Lipid measurements were done using Nile Red dye. It is a lipid-soluble fluorescent probe that is intensely florescent in organic solvents and hydrophobic environments but has a low quantum yield in water. Briefly, 250 µL of algal cell suspension was diluted to 1 mL and 4 µL of Nile Red solution in acetone (250 mg/mL) was added. The mixture was vigorously agitated on a vortex mixer and incubated in dark at room temperature for 10 min. Flourimetric analysis was performed using a PerkinElmer fluorescence spectrophotometer LS55, excitation and emission wavelengths were 490 nm and 585 nm, respectively. Both the excitation and emission slits were set to be 5 nm. The relative fluorescence intensity was calculated by subtraction of the auto-fluorescence of algal cells and the fluorescence intensity of Nile Red alone in the media [28,29].

### 2.7. Membrane damage

Effect of MNPs on the microalgal membrane integrity was evaluated by measurement of protein leakage and diffusion of nucleic acids at 3 days intervals [30,31]. After exposure with different concentrations of MNPs, the samples were centrifuged (13,000 rpm for 10 min) and supernatant was used to assay protein and nucleic acid content. Released proteins were quantified using Bradford micro-assay test against bovine serum albumin (BSA) standard curve [32]. The nucleic acids concentration was measured using Eppendorf BioPhotometer® D30.

### 2.8. Data analysis and statistics

All experiments were conducted in triplicates and results are presented as means ± standard deviation. Significant differences between control samples and MNPs exposed cells were determined by analysis of variance (ANOVA) followed by Tukey’s comparisons. The *p* value less than 0.05 was considered to be significant.

## 3. Results

### 3.1. Synthesis and characterization of magnetic nanoparticles

Injection of ammonium hydroxide to the iron solution resulted in a sudden change in the reaction color indicating the formation of magnetite nucleus. After drying, resulted particles were dark black with a metallic shine. FTIR spectra of L-lysine-coated magnetic nanoparticles are shown in Figure 1 (a1). Characteristic peaks of Fe-O appeared at 637.2 cm^−1^, 593.3 cm^−1^ and 450.5 cm^−1^. Peaks, due to OH groups on the surface of magnetite nanoparticles, appeared at 1629.5 cm^−1^ (deforming) and 3419.3 cm^−1^ (stretching). Amino acids NH stretching vibration overlaps with OH stretching vibration and C = O stretching vibration peak overlaps with OH deforming. FTIR diagram of pure L-lysine is provided in Figure 1(a2). In comparison with pure amino acid, shortening of the carboxyl group’s peak in Figure 1(a1) is due to the interaction with OH groups at the surface of nanoparticles. The saturation magnetization (Ms) values read from the magnetization plots was found to be 42 emu/g. Crystal structure of synthesized nanoparticles was analyzed using XRD in the range of 10 to 90 degrees of 2 theta angel. X-ray powder diffraction pattern of the nanoparticles is demonstrated by the characteristic features of magnetite, having intensity peaks at values expressed in 2θ degrees of 30, 35.5, 43, 57, and 63 (Figure 1b). Results of saturation magnetization analysis are shown in Figure 1c. No hysteresis was seen and magnetization curves are completely reversible, exhibiting the superparamagnetic behavior of the sample particles. DSC curve of MNPs is shown in Figure 1d. An endothermic peak, due to oxidation and change in crystallinity of magnetite (Fe_3_O_4_) crystals, was observed at 195.1°C. The next thermal change occurred at 384.3°C by decomposition of amino-acid coating.

**Figure 1.** Characterization of manufactured nanoparticles, FT-IR spectra of MNPs (a1) and L-lysine (a2), XRD pattern of MNPs indicating characteristic pattern of magnetite crystals (b), VSM diagram of the MNPs indicating superparamagnetic property (c), and DSC curve of MNPs indicating nanoparticles oxidation at 195.1°C and L-lys decomposition a 384.3°C (d).

Visual appearance of the nanoparticles was evaluated by TEM analysis. Micrographs revealed that the particles were spherical in shape with 4–10 nm in diameter and mean diameter of 7 nm (Figure 2(a, b)).

**Figure 2.** TEM Micrograph of the MNPs (a) and corresponding particle size distribution histogram (b).

### 3.2. Interaction of MNPs with C. vulgaris cells

Precise investigations were performed by SEM to visualize the potential of MNPs to interact with *C. vulgaris* cells and resulted micrographs are depicted in Figure 3. Comparing micrographs of untreated and treated cells revealed that nanoparticles can entrap *C. vulgaris* cells. It is obvious that MNPs can attach to the surface of microbial cells via nonspecific interactions such as electrostatic forces, hydrogen bonds, hydrophobic, and hydrophilic attractions [33]. Magnetic property and tendency of MNPs to agglomerate resulted in the clustering of attached cells between the particles [34]. This phenomenon was also observed via optical microscopic evaluations (Figure 4). At low concentrations of magnetic nanoparticles (below 100 µg/mL) cells were seen separately. By an increase in the nanoparticles concentration, obvious agglomerations can be observed that are made by interactions of magnetic nanoparticles with *C. vulgaris* cells.

**Figure 3.** SEM micrographs of *C. vulgaris* (a) and MNPs treated cells (b).

**Figure 4.** Microscopic appearance of the *C. vulgaris* cells exposed to various concentrations of MNPs (a: 0, b: 25, c: 50, d: 100, e: 200, f: 400, g: 600, and h: 800 µg/mL), increase in nanoparticles concentration resulted in the cells agglomeration.

### 3.3. Effects of MNPs on the cells growth rate

Growth curves of *C. vulgaris* cells in various concentrations of MNPs are depicted in Figure 5. The growth inhibition percentage (I%) of different concentrations of MNPs over 12 days are depicted in Figure 6. Low concentrations of MNPs promoted the growth of microalgal cells and minus values obtained for I%. However, a dose-dependent increase in I% was seen at concentrations higher than 25 µg/mL of IONs. Immense growth inhibition was observed at 600 and 800 µg/mL of MNPs with 64.7% and 96.3% growth inhibitions, respectively (Figure 6).

**Figure 5.** Growth curves of *C. vulgaris* cells at various concentrations of MNPs.

**Figure 6.** Growth inhibitory effects (I%) of MNPs on *C. vulgaris* cells over 12 days exposure.

### 3.4. Mitochondrial activity

Incubation of microalgae cells with MTT solution resulted in a change in cells color from green to dark blue. The blue formazan was clearly discernible in cell pellet and cells cytoplasm (Figure 7). In contrast to control samples, exposure of *C. vulgaris* cells to low concentrations of MNPs resulted in more MTT reduction (Figure 8). These results are in agreement with direct cell count results, which indicates the growth promotion effects of MNPs at lower concentrations. At initial days of exposure to ≥50 µg/mL MNPs, the mitochondrial activity reduced to 60%. By comparing the M% and I% results, it can be concluded that MNPs concentrations within the range of 50 to 400 µg/mL impaired the mitochondrial activity rather than killing the cells. This shows that microalgae can overcome this mitochondrial toxicity over time and by day 12, no significant reduction in mitochondrial activity was measured within the range of 50 to 400 µg/mL IONs.

**Figure 7.** Cell pellet (a) and microscopic appearance (c) of C. vulgaris cells in contrast to MTT treated cells (b and d).

**Figure 8.** Mitochondrial activity (M %) of C. vulgaris cells exposed to various concentrations of MNPs for 12 days.

### 3.5. Chloroplasts activity

The impact of MNPs on the *C. vulgaris* chloroplasts was evaluated by chlorophyll and carotenoids content assay (figure 9a, 9b, 10). Except the slight increase in chlorophyll and carotenoids by exposure to less than 25 µg/mL nanoparticles, higher concentrations of nanoparticles can reduce the chloroplasts activity to below 50%, during 6 days of exposure. *C. vulgaris* can overcome toxic effects of MNPs on chloroplasts within the range of 50 to 100 µg/mL and to some extent, 200 µg/mL by day 12.

**Figure 9.** Chlorophyll a content (a), and Chlorophyll b content (b) of *C. vulgaris* cells exposed to various concentrations of MNPs.

**Figure 10.** Carotenoids content of *C. vulgaris* cells exposed to various concentrations of MNPs.

### 3.6. Lipid content

The accumulation of lipid in *C. vulgaris* was monitored over 12 days as a function of time and nanoparticles concentration. The lipid content of MNPs exposed cells was compared to control cells. As can be concluded from Figure 11, significant reduction in lipid content was observed at ≥100 µg/mL MNPs on day 3. Whereas on day 6, lipid content reduction was significant at ≥200 µg/mL MNPs. Exposure to nanoparticles gradually induced cellular adaptation to higher concentrations and the effective concentrations were increased to ≥400 µg/mL on days 9 and 12. Some negative values are not statistically significant (p < 0.05) and can be due to experimental or instrumental errors.

**Figure 11.** Lipid content of *C. vulgaris* cells exposed to various concentrations of MNPs.

### 3.7. Membrane damage

Effects of MNPs on the microalgal membrane were studied as the function of protein leakage and nucleic acid diffusion. Throughout 12 days of experiment, an increase in the protein content was observed in all samples (Figure 12). But there was no significant (p-value >0.05) increase in the protein content due to the exposure to various concentrations of MNPs. Also, there was no detectable nucleic acid in the culture supernatants. Based on the results, MNPs have no extreme destruction effect on the *C. vulgaris* membrane integrity.

**Figure 12.** Released protein from *C. vulgaris* cells exposed to various concentrations of MNPs.

## 4. Discussion

Microbial cell wall is abundant with adhesion factors which facilitate the attachment of the cell to the surfaces. In the case of interaction of microbial cells with nanoparticulate materials, these materials are much smaller than the cell and so the adhesion factors act in a reverse form and became potential sites for attachment of nanoparticles. This phenomenon is reported for a wide variety of cells such as bacteria, yeasts, and algae which is the base of magnetic immobilization and magnetic harvesting [5,9,11]. In this experiment, the potential of MNPs to attach onto microalgal cells and developing agglomerated structures between the cells and MNPs was visualized in SEM micrographs. The hetero-agglomerations of algal cells and MNPs were also observed by an optical microscope. The attraction between attached microalgal cells and formation of hetero-agglomeration structures can also trigger and develop through other metallic and nonmetallic nanoparticles such as Al_2_O_3_, ZnO, Co_3_O_4_, CuO, TiO_2_, and SiO_2_ [35–37].

Attachment of nanoparticles to the cells surface has some effects on cells growth and proliferation [25,37]. This effect is deemed as concentration dependent. Meanwhile, high concentration of MNPs exhibits growth inhibitory effects, MNPs can act as iron supplement and at low concentrations promote cells growth and proliferation. In the current experiment, low concentrations of MNPs (≤25 µg/mL) stimulated the growth of algal cells and I% were obtained in minus value. However, this growth promotion effect was not significant (*p*> 0.05). These data indicated that *C. vulgaris* cells can tolerate magnetic nanoparticles in concentrations less than 400 µg/mL. Previous investigations indicated that these concentrations of magnetic nanoparticles are sufficient for effective magnetic immobilization and separation of the cells [9,38]. So, magnetic immobilization can be employed for immobilization of *C. vulgaris* cells without significant effects on the cells growth and population.

MNPs have also toxic effects on the cell organelles. These particles cause structural damage and depolarization in the mitochondria which leads to the loss of mitochondrial membrane potential, permeability transition (PT) pore, and cell death [39]. In this experiment, MTT assay was used to examine the impacts of MNPs on *C. vulgaris* mitochondrial activity [40–42]. Results were in close agreement with previous reports for toxic effects of MNPs on mitochondria [39]. Interestingly, mitochondria were even sensitive to low concentrations that have not significant effect on the cell growth. At initial days of exposure to MNPs, about 40% reduction in mitochondria activity was occurred at concentrations ≥50 µg/mL. Whereas significant reduction in the cell population was observed at concentrations ≥400 µg/mL. These findings indicate that MNPs in the concentration range from 50 to 400 µg/mL impaired the mitochondrial activity rather than cells death.

Impacts of MNPs on the other vital organelle, chloroplasts, were also evaluated by chlorophyll and carotenoids content assays. Chlorophyll a and chlorophyll b are the main chlorophylls in unicellular algae. Their concentrations are related to the level of chloroplasts activity and rate of photosynthesis. As observed for mitochondria, MNPs at concentrations higher than 50 µg/mL reduced chlorophyll and carotenoids content through 6 days exposure (*p*< 0.05). Chen *et al*. reported that the chlorophyll concentration in *C. vulgaris* cells that exposed to MNPs was decreased as a function of nanoparticles concentration. The significant reduction in chlorophyll concentration, however, is reported to occur in the presence of 200–1600 μg/mL of nanoparticles. Also, a decrease in CO_2_ absorption and photosynthetic rates was reported by increasing the MNPs concentration [43]. Chen *et al*. have used MNPs with 25 to 55 nm size distribution [43]. While, the particles diameter in the current study was ranged from 4 to 10 nm with the mean particle size of 7 nm [15–17]. Toxicological studies have shown that the size of the nanoparticles plays an important role in cytotoxicity [39,44,45].

It is believed that cell membrane damage is the primary mechanism through which nanostructures induce cytotoxicity [46]. MNPs can cause large aberrations in the cell membrane, with bubble-shaped protrusions extending from the cell body [47,48]. Nanoparticles can also penetrate into the phospholipid bilayer and disturb membrane integrity by inducing pore formation [46]. Pore formation in the plasma membrane can increase the membrane permeability. This effect was reported for both animal and microbial cells, *e.g*. A549 lung carcinoma cells, microvascular endothelial cells, and *Rhodococcus erythropolis*, but not for all cells [2,49,50]. For instance, investigations on the microvascular endothelial cells showed that MNPs do not significantly affect membrane permeability [51]. Particularly in the case of *C. vulgaris*, MNPs have induced no significant membrane damage. Interactions of nanoparticles with cell membrane are affected by the physicochemical characteristics of nanoparticles. It has been suggested that size, morphology, and surface coating of nanoparticles are the major parameters affecting the nanoparticles and cells interactions [52].

## 5. Conclusions

MNPs have the potential to cause toxicity in microalgal cells. Toxicity to cell organelles, mitochondria and chloroplasts, was observed in algal cells exposed to high concentrations of MNPs. After more than 6 days of exposure to stress generating concentrations of MNPs, it was found that microalgae could overcome the resulted damages. Therefore, in the aspect of the biotechnological process and environmental concerns caused by long-term exposure to MNPs, harmful toxic effects should only be expected during the initial days and at high concentrations. The present study reveals that the effect of MNPs on the growth and metabolic status of *C. vulgaris* is critically dependent on the concentration of MNPs and exposure time.

## Data Availability

Impacts of magnetic nanoparticles on the *C. vulgaris* cells were investigated. Growth inhibitory effect was seen at concentrations ≥400 µg/mL. Significant effects on chloroplast and mitochondrial activity occurred at ≥50 µg/mL. Microalgal cells could overcome the imposed damages after certain days.

## Data Availability Statement

Data available on request from the authors.
